# The miR-302/367 cluster: a comprehensive update on its evolution and functions

**DOI:** 10.1098/rsob.150138

**Published:** 2015-12-02

**Authors:** Zeqian Gao, Xueliang Zhu, Yongxi Dou

**Affiliations:** State Key Laboratory of Veterinary Etiological Biology, Key Laboratory of Veterinary Parasitology of Gansu Province, Lanzhou Veterinary Research Institute, Chinese Academy of Agricultural Sciences, 1 Xujiaping, Yanchangbu, Lanzhou, 730046 Gansu, China

**Keywords:** miR-302/367 cluster, evolution, transcriptional regulation, cell cycle, cellular signalling, epigenetic regulation

## Abstract

microRNAs are a subclass of small non-coding RNAs that fine-tune the regulation of gene expression at the post-transcriptional level. The miR-302/367 cluster, generally consisting of five members, miR-367, miR-302d, miR-302a, miR-302c and miR-302b, is ubiquitously distributed in vertebrates and occupies an intragenic cluster located in the gene *La-related protein 7* (*LARP7*). The cluster was demonstrated to play an important role in diverse biological processes, such as the pluripotency of human embryonic stem cells (hESCs), self-renewal and reprogramming. This paper provides an overview of the mir-302/367 cluster, discusses our current understanding of the cluster's evolutionary history and transcriptional regulation and reviews the literature surrounding the cluster's roles in cell cycle regulation, epigenetic regulation and different cellular signalling pathways.

## 1. Introduction

The first animal microRNA (miRNA), lin-4, was discovered in *Caenorhabditis elegans* and was found to be involved in coordinating development timing via post-transcriptional regulation of a protein-coding gene, *lin-14* [1,2]. Since then, numerous miRNA genes have been predicted and identified in animals, plants and viruses [3–6].

The miRNA-mediated silencing mechanism executes important regulatory functions in plants and animals [7]. In animals, primary miRNA transcripts (pri-miRNAs) are generated from single or clustered miRNA genes and sequentially undergo two consecutive processing steps by Drosha and Dicer, two members of the RNase Ш endonuclease family, to give rise to approximately 22 bp miRNA-harbouring duplexes [8,9]. Once loaded onto the small RNA-induced silencing complex (RISC), one of the strands, mature miRNA, is retained and serves as a guide to target transcripts via imperfect sequence complementarities with the sites mostly located in the 3′UTR of mRNAs, leading to target transcript degradation or translational repression [10,11]. Although the level of inhibition employed by miRNAs is relatively modest, resulting in only minor adjustments in protein output [12,13], their regulatory action is important in nearly all aspects of biological activities [14–18].

miRNA genes are distributed in diverse genomic locations, including intergenic regions, introns/exons of protein-coding genes and non-coding RNA genes. Intriguingly, while most miRNAs are expressed individually and scattered across the entire genome, a portion of them is clustered and expressed as polycistronic precursors. According to miRBase, more than a quarter of both fruitfly and human miRNA genes are less than 10 kb away from other miRNA loci [19]. The majority of these clustered miRNA genes are co-expressed and show a higher degree of evolutionary conservation [20]. The miR-302/367 cluster is highly conserved and vertebrate-specific. The cluster was initially identified to be specifically expressed in undifferentiated human embryonic stem cells (hESCs), and their malignant counterpart human embryonic carcinoma cells (hECCs), and was indicated to play a role in maintenance of pluripotency of stem cells and cancer formation [21,22]. Accumulating evidence demonstrates that the miR-302/367 cluster plays significant roles in regulation of cellular proliferation, differentiation and reprogramming. Herein, we review the current understandings to date as to the roles of its members in a diverse range of biological processes.

## 2. Molecular characteristics of the cluster

The miR-302/367 cluster gene was found to be located in an intron on the 4q25 region of human chromosome 4, and transcribed by RNA polymerase II (Pol-II) to generate a capped and polyadenylated miRNA precursor that possessed eight miRNAs: miR-367, 302d, 302c-5p, 302c-3p, 302a-5p, 302a-3p, 302b-5p and 302b-3p [23]. miR-367 was slightly different in the seed sequence from miR-302a–302d, but they shared a portion of common mRNA targets. Interestingly, the 3′UTRs of upregulated transcripts in Dicer-null ESCs were shown to be enriched for the ‘GCACUUU’ and ‘AGCACUU’ motifs, complementary to the miR-302 family seed sequence, indicating the importance of the miR-302 family in the regulatory network in ESCs [24,25].

The starting point of comparative genomic analysis of the mir-302/367 cluster was the retrieval of mir-302 members and mir-367 precursor sequences. A combined searching strategy was undertaken to identify mir-302/367 family members in multiple genomes from Ensemble Genome Database (http://www.ensembl.org/). For some well-annotated genomes, mir-302 sequences were directly extracted from the database. Additionally, BLAST searches [26] were performed to identify the homologous sequences. The investigated species in this study were several representing vertebrate species, including *Petromyzon marinus* (jawless fish), *Danio rerio* (bony fish), *Xenopus tropicalis* (amphibian), *Ornithorhynchus anatinus* (ancient mammal), *Homo sapiens* (primate), *Dasypus novemcinctus* (reptile) and *Gallus gallus* (bird). The results revealed that the miR-302/367 cluster is conserved among vertebrates, but the copy number and genomic location of the cluster gene vary. As shown in figure 1*a*, the ancient vertebrate *P. marinus* contains only one copy of miR-302 members. No member of the miR-302/367 cluster has been discovered in bony fish such as *D. rerio*, most probably owing to the loss of this cluster during the evolutionary process. However, according to multiple sequence alignment, we found that the mir-302 of *P. marinus* (pma-mir-302) was not contained in the mir-302/367 family. pma-mir-302 only shared the seed sequence of the 3′ mature miRNAs with the 3′ mature sequence of the mir-302/367 family (figure 1*b*). It did not share the 5′ mature miRNA nor the precursor sequence [27]. The fact that no homologue can be found in jawless fish and bony fish suggested the emergence of mir-302/367 at the branch leading to the tetrapoda. The whole genome of the amphibian *X. tropicalis* codes two miRNAs, miR-302 and miR-367, located in the intron of the *LARP7* gene. Higher vertebrates such as mammals, birds and reptiles commonly possess ‘classical’ structure, including four miR-302 members and one miR-367, in the cluster locus. Interestingly in primates, besides the four members of miR-302, there also exist another two miR-302 members, namely miR-302e and miR-302f, which are both intergenic miRNAs and located in chromosome 11 and 18, respectively. It was also observed that the seed sequence of *Gallus gallus* miR-1811, a bird-specific miRNA located in the miR-302/367 cluster gene locus, shows a high similarity to miR-367, indicating that miR-1811 might have been generated by tandem duplication of miR-367. The expansion or shrinking of the miR-302 family by tandem duplication or deletion generated miR-302/367 clusters of different lengths in different species. The RNA sequencing data from *H. sapiens* and *Mus musculus* confirmed that the 3′ arm is highly expressed and more conserved compared with the 5′ arm in most miR-302 family members (figure 1*c*) [28–30].

**Figure 1.** (*a*) Phylogenetic tree of vertebrate species and genomic organization of miR-302 and miR-367 sequences. Red arrows depict miR-302 family members, green arrows depict miR-367, black arrow depicts pma-miR-302 and blue arrow depicts bird-specific miR-1811 sequence. Arrows linked by the same straight line indicate miRNAs linked in the genome by less than 10 kb. (*b*) Multiple sequence alignment of miR-302 precursor sequences. (*c*) Consensus structure of the miR-302 precursor in vertebrates, coloured according to sequence conservation.

miRNAs have evolved to target a diverse range of transcripts by mechanisms including seed shifts, insertions and nucleotide editing, generating different seed sequences and hence altering the profile of targeted transcripts [31,32]. Another mechanism changing miRNA target specificity is arm switching [33]. Whereas most mature miRNAs from the miR-302 family generally originate from the 3′ arm of the hairpin precursor, a small quantity of mature miR-302 members are derived from the opposite arm. For instance, the miR-302e hairpin precursor of humans predominantly generates mature miRNAs from the 5′ arm [34]. Most importantly, the sequences of mature miRNAs produced by arm switching have been demonstrated to regulate a distinct set of targeted transcripts and, ultimately, result in the alteration of the cellular regulatory network [35].

## 3. Transcriptional regulation of the cluster

Intergenic miRNA genes were believed to possess their own transcriptional units, whereas intronic miRNAs were more likely transcribed with their host genes [36]. The miR-302/367 cluster, composed of several intronic miRNAs, was initially proposed to be transcribed with their host gene *LARP7*. However, a recent study disclosed that the cluster contains its own transcriptional unit [23]. The intact sequence of the polycistronic miRNA gene possesses the classical sequence motifs for TATA box and polyadenylation signal. The primary transcript is a 1974 nt long RNA with the 5′ end located 153 nt upstream from the first encoded miRNA (miR-302b-5p), and the 3′ end sited approximately 12 nt downstream from a classical polyadenylation signal (figure 2*a*) [23,37].

**Figure 2.** (*a*) The transcriptional factors and main targets of the miR-302/367 cluster. The transcriptional regulators in the left upper corner have been functionally validated; dark arrows depict upregulation; black lines indicate repression. TFs in the right upper corner were newly identified by the ENCODE project and the relationship of most of them to the miR-302/367 cluster is putative. (*b*) Proposed mechanism of miR-302 members' mediation of cell cycle regulation.

After identification of the gene structure of the miR-302/367 cluster by means of 5′ RACE assay, 3′ RACE assay and sequence alignment, several transcriptional factors (TFs), Oct3/4, Cdx2, Sox2, Rex1 and Nanog, were predicted to be capable of targeting the promoter of the cluster using bioinformatic methods [23]. It was experimentally demonstrated that Oct3/4, Nanog, Rex1 and Sox2 act as transcriptional activators of the miR-302/367 cluster [37,38]. More specifically, the two putative binding sites of Sox were located in the exon 1 and intron 1 of *LARP7*, respectively [23]. Furthermore, CHIP assays revealed a physical interaction between Sox2 and the binding sites [38], verifying that Sox2 is the upstream regulator of the miR-302/367 expression. Using similar experimental approaches, Gata6 was identified as a new transcriptional regulator to activate the expression of miR-302/367 cluster in mouse embryos [39,40]. There also exist some cofactors of TFs that facilitate the transcriptional activation of the cluster. One publication showed that hyaluronan-induced CD44v3 (a hyaluronan receptor) interaction with Oct4–Sox2–Nanog increases the transcriptional level of the cluster [41]. In addition, some regulators could indirectly affect the transcriptional level of the miR-302/367 cluster via a diverse range of signalling pathways. For instance, the transcription of the cluster was regulated by the Wnt/*β*-catenin pathway and bone morphogenetic protein (BMP) signalling pathway [42,43]. A recent study has also revealed that an anti-allergy drug, tranilast, promoted miR-302 members expression through binding to the two aryl hydrocarbon receptor binding motifs in the promoter [44].

Additional information on transcriptional regulation became accessible through the recent release of data from the encyclopaedia of DNA elements (ENCODE) project [45]. ENCODE's results uncovered 1292 TF–miRNA interactions (transcriptional factors regulate miRNAs' expression) and 421 miRNA–TF interactions (transcriptional factors' expression regulated by miRNAs), in turn suggesting tightly coupled autoregulatory loops involving miRNAs and TFs. Of the 118 TFs, seven pertained to the miR-302/367 cluster, including the previously known Oct 3/4 and 6 novel TFs (figure 2*a*).

## 4. Biological functions of the miR-302/367 cluster

Cyclin D1 and CDK4 were the first miR-302/367 targets identified, by means of reporter assays [38,46]. Henceforward, numerous targets of miR-302/367 cluster have been identified. The majority of the cluster target genes (figure 2*a*) can be classed into three groups depending on their functions. To begin with, the miR-302/367 cluster was found to be involved in regulating cell signalling pathways, including TGF-*β*/Nodal signalling, PI3K–AKT signalling and BMP signalling, by directly repressing expression of some key components in the pathways [24,37,47]. Furthermore, a large proportion of those target genes are involved in regulating the cell cycle of stem cells or carcinoma cells. The remaining verified targets of miR-302/367 are key mediators of a diverse range of processes, including epigenetic regulation and glucose metabolism. The miR-302/367 cluster, specifically expressed in embryonic stem cells, induced pluripotent stem cells (iPSs) or tumour cells, represses the targets mentioned above, to coordinate proliferation, differentiation, pluripotency maintenance and reprogramming.

### 4.1. Roles in cell cycle regulation

The decision to be quiescent or resume activity in somatic cells is dictated by extracellular and intracellular stimuli [48,49]. Proliferation of animal cells requires overcoming the G1-to-S restriction (R) point, which is a key step for cell cycle progression, and relies largely on regulation of retinoblastoma (RB) protein activity [50]. RB without linking phosphate groups can sequester the TFs of E2F and prevent them from activating the transcription of target genes. RB is phosphorylated owing to stimulation by mitogenic signals, resulting in its inactivation and consequently permitting progression through the cell cycle. Completion of phosphorylation of RB (pRB) needs two steps [51,52]. First, cyclin D combines with CDK4 and CDK6, resulting in pRB, partial release of the E2F factors and activation of their downstream target genes *Cyclin E* and *Cdc25A*. Subsequently, Cdc25A removes phosphate groups from CDK2, facilitating it to combine with Cyclin E and further phosphorylate pRB to achieve full release of E2F factors and progression from G1 into S phase. Compared with somatic cells, ESCs do not possess an R point, allowing the rapid progression through G1 even in the absence of growth signals. On account of the absence of CDK inhibitors in ESCs, active Cyclin E/CDK complex is maintained at high levels and results in a constitutively hyperphosphorylated pRB and transcription of E2F targets [25].

The first discovery revealed that miRNA-deficient ESCs accumulated at G1, indicating that miRNAs are also a part of the network that regulates the G1-to-S transition [53,54]. Increasing evidence has directly demonstrated that the members of the miR-302/367 cluster play a critical role in regulation of the balance of G1-to-S transition. CDKN1A (cyclin-dependent kinase inhibitor 1, also known as p21), which was referred to as an inhibitor to Cyclin E/CDK2 complex, was the first verified target of the miR-302/367 cluster [55,56]. miR-302 members directly silenced the expression of CDKN1A and hence augmented the abundance of Cyclin E/CDK complex, promoting the transition of mouse embryonic stem cells from G1 to S phase [56]. However, a subsequent publication revealed that miR-302 members could inhibit human pluripotent stem cell proliferation by enhancing multiple G1 phase arrest pathways [57]. Three target genes were identified: CDK2, Cyclin D1/D2 and BMI1 polycomb ring finger oncogene (BMI-1) [46,57]. miR-302 members strongly suppress BMI-1 to stimulate CDKN2A (cyclin-dependent kinase inhibitor 2A, or p16) expression, thus giving rise to decrease in the output of CDK4/6 and Cyclin D complex and finally repressing the G1-to-S transition. miR-302 members also can directly inhibit the expression of Cyclin D1/2, CDK2 and ARID4a (AT-rich interacting domain 4a, also known as RBP1), which represses the phosphorylation of pRB, leading to failed expression of cell cycle genes and cellular G1 phase arrest (figure 2*b*) [57,58]. In addition, miR-302 members can mediate other pathways to regulate the cell cycle via targeting the transcripts of epidermal growth factor receptor (*EGFR*), C–C chemokine receptor type 5 (*CCR5*), C–C motif ligand (*CCL5*) and C–X–C chemokine receptor type 4 (*CXCR4*) [58–60].

### 4.2. Roles in epigenetic modification

miR-302 members can target different epigenetic factors resulting in global demethylation in target cells [61]. DNA demethylation typically appears after fertilization at the one- to eight-cell stage or a few days after the development of primordial stem cells [62,63]. In the zygote, global demethylation was shown to occur at the promoter binding region of several ESC-specific TFs. Indeed, miR-302 members repressed lysine-specific histone demethylase 1 and 2 (AOF1 and AOF2) and methyl-CpG binding proteins (MECP1 and MECP2), leading to destabilization of DNA methyltransferase 1 which is involved in genome-wide demethylation and consequently promotes reprogramming and iPS cells development [64]. In addition, a recent study has identified a new epigenetic suppressor, methyl-DNA binding domain protein 2 (MBD2), which blocked full reprogramming of somatic to iPS cells via directly binding to Nanog promoter elements to prevent transcriptional activation. Overexpression of the miR-302/367 cluster significantly increased the conversion of reprogrammed iPS cells by repressing MBD2 expression, thereby augmenting Nanog expression [65].

### 4.3. Roles in cellular signalling

The miR-302/367 cluster has been demonstrated to be involved in regulation of various cellular signalling pathways, such as the BMP signalling pathway and TGF-*β*/Nodal/Smad-2/3 pathway, to coordinate different biological processes. More specifically, miR-302 members can fine-tune stem cell self-renewal through promotion of BMP signalling. Three BMP inhibitors, TOB2, DAZAP2 and SLAIN1, were silenced via binding of mature miR-302 members to the 3′ UTRs of their transcripts, leading to repression of stem cell differentiation and maintenance of stem cell pluripotency [66]. Another study found that the miR-302/TGF-*β*/Nodal/Smad-2/3 pathway was also involved in epithelial–mesenchymal transition (EMT). EMT is a form of epithelial plasticity that is essential for normal embryonic development. In EMT, epithelial cells, which form monolayers that line many body structures and compartments, disintegrate attachments to neighbouring cells, and display elongated morphology and enhanced motility [67]. miR-302 members directly repressed the expression of the transforming growth factor beta receptor 2 (TGFBR2), and Ras homologue gene family, member C (RHOC) genes, resulting in facilitation of EMT [68,69]. Silencing the expression of TGFBR2 and RHOC by small interfering RNAs has been shown to facilitate the conventional reprogramming of somatic cells which were induced using the four classical TFs [69]. In addition, miR-302 members could negatively regulate the level of Lefty1 and Lefty2 (Nodal inhibitors), and thus became upstream modulators of the TGF-*β*/Nodal signalling pathway, striking a balance between pluripotency and differentiation [70].

## 5. Concluding remarks

The miR-302/367 cluster is widely distributed in vertebrates and plays vital roles in cellular self-renewal, differentiation and reprogramming, mainly through targeting the key genes in cell cycle regulation, cellular signalling regulation and epigenetic regulation. The role of the miR-302/367 cluster is expanding. The cluster can also fine-tune stem cell proliferation or differentiation through other pathways, for example regulation of glucose metabolism and endoplasmic reticulum homeostasis [71,72]. The miR-302/367 cluster regulates the pathways through silencing key components, and the feedback of the regulated pathways can impact the expression of the cluster. Most recent publications on miR-302 members have supported a positive correlation between miR-302/367 upregulation and BMP signalling promotion. Another positive feedback loop is also composed of the cluster and its TFs, such as Oct4. These regulatory networks are important for us to understand and control the physiological state of cells. Increasing studies in the future will provide us with a clear mechanism by which miR-302 members fulfil the cellular self-renewal, differentiation and reprogramming in a more integrated network.

## Data accessibility

mir-302 precursor sequences: miRBase accessions MI0000738, MI0000772, MI0000773, MI0000774, MI0001211, MI0003700, MI0003701, MI0003702, MI0004878, MI0017123, MI0006903, MI0006904; Ensemble Genome Browser accessions ENSDNOG00000038602, ENSDNOG00000043944, ENSDNOG00000027052, ENSDNOG00000026812, ENSDNOG00000017050, ENSDNOG00000016990.
